The article "Prognostic Comparison between cTACE and H101-TACE in Unresectable Hepatocellular Carcinoma (HCC): A Propensity-Score Matching Analysis" was retracted in 2023. Reasons: signs of a paper mill; suspected computer-generated content; unreliable results or conclusions; lack of ethics approval or compliance.

# Prognostic Comparison between cTACE and H101-TACE in Unresectable Hepatocellular Carcinoma (HCC): A Propensity-Score Matching Analysis

**DOI:** 10.1155/2022/9084852

**Published:** 2022-09-02

**Authors:** Man Yao, Simo Cheng, Xiaofeng Zhai, Hetong Zhao, Jing Hong, Xiaoyan Li, Yongbin Meng, Wei Chen

**Affiliations:** ^1^Department of Integrative Oncology, The First Affiliated Hospital of Navy Military Medical University, Shanghai 200433, China; ^2^School of Traditional Chinese Medicine, Navy Medical University, Shanghai 200433, China; ^3^Department of Radiology, The First Affiliated Hospital of Navy Military Medical University, Shanghai 200433, China

## Abstract

**Background:**

Transarterial chemoembolization (TACE) is the most common treatment for patients with HCC who are unsuitable for radical therapies. Conventional TACE (cTACE) takes advantage of the preferential hepatic arterial supply of HCC for the targeted delivery of chemotherapeutic agents suspended in lipiodol, followed by embolization or reduction of arterial flow using various types of particles while sparing the surrounding liver parenchyma. *Aims and Objectives*. The current study is aimed at comparing the efficacy and safety profiles of transarterial infusion of recombinant human type-5 adenovirus (H101-TACE) with conventional transarterial chemoembolization (cTACE) in patients with unresectable hepatocellular carcinoma (HCC).

**Methods:**

Unresectable HCC patients that received H101-based TACE or cTACE from August 2018 to September 2021 were retrospectively evaluated. Propensity score matching (PSM) has a 1 : 1 ratio to eliminate possible confounder imbalances across cohorts. The main outcome was overall survival (OS), while secondary outcomes were progression-free survival (PFS) and tumor response.

**Results:**

This study included 111 patients classified across two cohorts: the H101-TACE cohort (*n* = 37) and the cTACE cohort (*n* = 74). Median OS within the H101-TACE cohort was 9.0 months longer than within the cTACE cohort before PSM (22.1 vs. 13.1 months, *P* = 0.043) and 9.3 months longer following PSM (22.1 vs. 12.8 months, *P* = 0.004). The median PFS within the H101-TACE cohort was 3.2 months longer compared to the cTACE cohort before PSM (6.5 vs. 3.3 months, *P* = 0.046) and 2.5 months after PSM (6.5 vs. 4.0 months, *P* = 0.012). The disease control rate for H101 and control cohorts was 81.1% and 59.5%, accordingly (*P* = 0.039).

**Conclusion:**

The present study demonstrated that the H101-TACE is safe and efficient and can considerably enhance prognostic results for unresectable HCC compared to cTACE.

## 1. Introduction

Hepatocellular carcinoma (HCC) is the seventh-most prevailing cancer globally and the second most prevailing driver of tumor-associated [1]. In China, many cases of advanced HCC were confirmed, having lost the chance of surgical resection [2]. It remains debatable regarding the selection of the ideal chemotherapy drug in TACE for unresectable HCC. Up to now, agents typically employed for TACE chemotherapeutics remain 5-fluorouracil, oxaliplatin, or pirarubicin. Indications for these alternatives, such as H101, have not been determined. Consequently, productive TACE maintenance in such cases is still proving to be a great challenge [3].

The article "Prognostic Comparison between cTACE and H101-TACE in Unresectable Hepatocellular Carcinoma (HCC): A Propensity-Score Matching Analysis" was retracted in 2023. Reasons: signs of a paper mill; suspected computer-generated content; unreliable results or conclusions; lack of ethics approval or compliance.

Oncolytic virus (OVs) therapy is highly novel and potentially effective approaches in antitumor therapies, which can selectively infect and kill cancer cells without harming the natural or recombinant viruses of normal cells [4–7]. Two approaches produce the OVs: directing blood-based antitumor immunity, targeted lytic effect on tumor cells, and selective replication within tumor cells [8–10]. Currently, many pre- and clinical settings are used to evaluate OVs such as adenovirus (Ad), herpes simplex virus (HSV), Newcastle disease virus (NDV), and measles virus [11]. A phase Ib trial in cases of advanced melanoma reported that oncolytic viral therapy enhances intratumoral T cell invasion and promotes anti-PD-1 immunotherapies [12]. Recombinant human adenovirus type 5 (H101, Oncorine), the world's first and the only oncolytic virus antitumor drug in China, was accepted by the State Medical Products Administration of China in treating advanced nasopharyngeal carcinoma in 2005 [10]. Several clinical trials have shown that H101 can treat head and neck cancer and bring certain clinical benefits to patients with other tumors (such as hepatocellular carcinoma, pancreatic cancer, and nonsmall cell lung cancer). Meanwhile, He and Lin [13] and Dong et al. [14] have shown that H101 together with TACE was a low-risk, efficacious therapeutic option that delays HCC development and prolongs survival in HCC cases.

Therefore, the current study compares the efficacy and safety characteristics of recombinant human type-5 adenovirus trans-arterial infusion (H101-TACE) with conventional transarterial chemoembolization (cTACE) in patients with unresectable hepatocellular carcinoma (HCC). We used propensity score matching (PSM) to reduce intercohort basal differences in this trial and compared OS, PFS, tumor response, and adverse events between the 2 groups.

## 2. Methods

### 2.1. Patient Selection

This is a retrospective cohort study in our hospital from August 2018 and September 2021. HCC was confirmed by either histology/radiology assessments depending on the Guidelines of the Chinese Society of clinical oncology (CSCO) [15]. Cases enrolled within this investigation attained inclusion criteria: (1) adult cases were staged as BCLC-B or BCLC-C as per BCLC protocol, (2) Child-Pugh grade A or B, and (3) Eastern Cooperative Oncology Group (ECOG) performance status of 0–2. Exclusion criteria consisted of [16] (1) combined with heart, brain, kidney, lung, and other organ diseases; (2) the formation of main portal vein cancer thrombus, bile duct cancer thrombus, and collateral vessel; (3) severe varices of gastric fundus and esophagocardia, severe portal hypertension, with the risk of rupture and bleeding; (4) systemic infection sepsis, liver abscess; (5) the liver function of patients were Child-Pugh grade C; (6) patients with severe cirrhosis; (7) tumor accounts for 70% or more of the whole liver; and (8) allergic constitution or allergic to the drugs involved in this study.

The article "Prognostic Comparison between cTACE and H101-TACE in Unresectable Hepatocellular Carcinoma (HCC): A Propensity-Score Matching Analysis" was retracted in 2023. Reasons: signs of a paper mill; suspected computer-generated content; unreliable results or conclusions; lack of ethics approval or compliance.

The study has been accepted by the Institutional Review Board of our hospital (no. CHEC2010-112) and follows the tenants of the Declaration of Helsinki.

### 2.2. Treatment Procedures

All cases underwent percutaneous femoral artery puncture by using the conventional Seldinger method. Epirubicin was used for cTACE. The dose of epirubicin and lipiodol depended on the accuracy of liver tumor position, tumor dimensions, and tumor quantity. In cases receiving H101-TACE, H101 was given following epirubicin administration via catheter into the hepatic artery feeding the tumor(s). Overall, 1.0 × 10^12^vp dissolved within 10 ml 0.9% sodium chloride injection. Aseptically purified particles of virus H101 for clinical use were manufactured by Shanghai Sanwei Biotech™ (China). The National Institute for the Control of Pharmaceutical and Biological Products (Beijing, China) evaluated potency, sterility, and overall safety profile. TACE protocols were conducted via in-patient strategy through an interventional radiologist with over TACE experience. The interval between TACE procedures was 1.5–3 months.

### 2.3. Drug Combinations

Across both cohorts, tropisetron was employed for emesis prophylaxis; rabeprazole sodium was employed for reducing gastric acid levels, with compound glycyrrhizin employed for hepatic protection. Additional symptomatic support therapies were additionally adopted.

### 2.4. Follow-Up

All clinical cases were assessed through computed tomography (CT) scan following the TACE session (one month) and were followed up post-TACE session until the mortality event or the final follow-up ended on December 6, 2021. Data on patients' condition/survival were recorded every 60 days. When progression was clinically ascertained, nonsurgical treatments like TACE, targeted drugs, PD-1/PD-L1, and traditional Chinese medicine were rapidly deployed, depending upon the overall condition, residual liver function, and individual case progression profile.

The article "Prognostic Comparison between cTACE and H101-TACE in Unresectable Hepatocellular Carcinoma (HCC): A Propensity-Score Matching Analysis" was retracted in 2023. Reasons: signs of a paper mill; suspected computer-generated content; unreliable results or conclusions; lack of ethics approval or compliance.

The main outcome included overall survival (OS), describing duration from the date of TACE until mortality event or final follow-up. Secondary outcomes were progression-free survival (PFS) and tumor responses. The PFS describes the timeframe from the treatment to disease progression, mortality event, or final day of follow-up. The modified Response Evaluation Criteria in Solid Tumors (mRECIST) was employed to assess the efficacy [17].

Hepatic function, hematologic system, and clinical symptom patterns of adverse events were evaluated during the 3rd and 5th day following TACE, in line with Common Terminology Criteria for Adverse Events (CTCAE) version 5.0.

### 2.5. Statistical Analyses

SPSS version 24.0 was used for statistical analyses. Pearson's *χ*^2^ test and independent *t*-test were employed for comparative analysis for correlations across differing variable types. Kaplan-Meier methodology was employed to determine survival curves, while the log-rank test assessed survival. Variables with a *P* value < 0.1 within the univariate analysis were included within multivariate Cox's proportional hazards regression model assessment for valuing parameters that influenced OS. *P* < 0.05 was considered statistically significant. PSM (propensity score matching) was conducted to minimize confounding influence and balance baselines across cohorts. A 1 : 1 match for TACE/H101-TACE cohorts was performed through nearest-neighbour methodology, using a calibre of 0.1. SM was performed through the MatchIt package (R software-package Version 4.1.3, R Development Team, Vienna, Austria). OS and PFS figures are made with GraphPad.

## 3. Results

### 3.1. Investigation Cohort Constitution/Clinical Profiles

Overall, 132 unresectable HCC cases underwent H101-TACE or cTACE were evaluated for eligibility. Finally, 111 cases participated in this investigation (37 within the H101-TACE cohort and 74 within the cTACE cohort) before PSM. Comprehensive essential case profiles before PSM are listed in Table 1. Apart from ALB (*P* = 0.043), two cohorts were comparable within demographic, clinical, and tumor characteristics (*P* > 0.05). Following PSM, 36 cases within the H101-TACE cohort and 36 cases within the cTACE cohort were present, accordingly, with most features equivalent across both cohorts (*P* > 0.05, Table 2).

### 3.2. Survival Analysis before/following PSM

Figure 1 highlights that the median OS period was 22.1 (95% CI: 12.58-31.62) months and 13.1 (95% CI: 10.99–15.11) months within H101-TACE and cTACE cohort, accordingly, with statistical significance confirmed for variations across both cohorts (*P* = 0.043, Figure 1(a)) Similarly, the median PFS period for the H101-TACE cohort was 6.5 months (95% CI: 4.92–8.09), significantly prolonged compared to the cTACE cohort (3.3 months, 95% CI: 2.30-4.36, *P* = 0.046; Figure 1(c)).

The article "Prognostic Comparison between cTACE and H101-TACE in Unresectable Hepatocellular Carcinoma (HCC): A Propensity-Score Matching Analysis" was retracted in 2023. Reasons: signs of a paper mill; suspected computer-generated content; unreliable results or conclusions; lack of ethics approval or compliance.

Following 1 : 1 PSM, H101-TACE cohort prognoses were also highly improved in comparison to cTACE cohort (OS: median OS time, 22.1 months, 95% CI: 12.58-31.62 vs. 12.8 months, 95% CI: 8.96-16.64, *P* = 0.004; Figure 1(b); for PFS: median PFS time, 6.5 months, 95% CI: 4.94-8.07 vs. 4.0 months, 95% CI: 4.94-8.07, *P* = 0.012; Figure 1(d)).

### 3.3. Generalized Risk Factors Linked to OS/PFS

Prior to PSM, Child–Pugh grade (HR = 2.018, 95%CI = 1.187–3.433), HBsAg (HR = 0.359, 95%CI = 0.111–1.157), AFP level (HR = 2.052, 95%CI = 1.192 − 3.534), tumor size (HR = 0.888, 95%CI = 0.521 − 1.515), tumor thrombus (HR = 6.911, 95%CI = 3.425 − 13.942), lymph node metastasis (HR = 2.322, 95%CI = 1.211 − 4.451), treatment option (HR = 0.544, 95%CI = 0.300–0.637), BCLC (HR = 2.999, 95%CI = 1.705 − 5.272), ECOG 1/0 (HR = 2.664, 95%CI = 1.520 − 4.669), and ECOG 2/0 (HR = 9.06, 95%CI = 2.673 − 30.705) were recognized as possible risk factors of OS (Table 3).Whereas HBsAg (HR = 0.173, 95%CI = 0.051–0.589), AFP level (HR = 1.923, 95%CI = 1.069 − 3.460), tumor thrombus (HR = 4.944, 95%CI = 2.300 − 10.628), ECOG 1/0 (HR = 2.300, 95%CI = 1.274 − 4.151), and ECOG 2/0 (HR = 7.408, 95%CI = 1.985 − 27.654) were independent risk factors for OS (Table 3).

AFP level (HR = 1.514, 95%CI = 0.995 − 2.304), lymph node metastasis (HR = 2.004, 95%CI = 1.083 − 3.708), treatment option (HR = 0.649, 95%CI = 0.423–0.0.996), and ECOG 2/0 (HR = 9.397, 95%CI = 2.750 − 32.107) were potential risk factors for PFS (Table 3). Meanwhile, AFP level (HR = 1.548, 95%CI = 1.009 − 2.374), ECOG 1/0 (HR = 1.207, 95%CI = 0.760 − 1.919), and ECOG 2/0 (HR = 10.713, 95%CI = 3.100 − 37.028) were independent risk factors of PFS (Table 3).

### 3.4. Tumor Response

The tumor responses were assessed in line with mRECIST (Table 4). Disease control rate (DCR) was described as the sum of CR + PR + SD. The DCR for the H101-TACE cohort and cTACE cohort was 81.1% and 59.5%, accordingly, with this variation having statistical significance (*P* = 0.039). The objective response rate (ORR) was calculated according to CR + PR. The ORR of the two cohorts was 62.2% and 36.5% (*P* = 0.018), respectively. A better response was indicated for the treatment based on H101, according to the significant difference between the two cohorts.

### 3.5. Adverse Events

Results showed that there was no statistical significance across both cohorts in liver function indexes and blood routine tests (*P* > 0.05, Table 5) except CRP on the 3rd day (*P* = 0.028). The incidence of liver pain (*P* > 0.05) and vomiting (*P* > 0.05) did not markedly vary across cohorts (Table 6). Pyrexia was recorded across both cohorts, with the H101-TACE cohort being markedly increased compared to the cTACE cohort, especially in grade 2 and grade 3 (*P* = 0.048).

The article "Prognostic Comparison between cTACE and H101-TACE in Unresectable Hepatocellular Carcinoma (HCC): A Propensity-Score Matching Analysis" was retracted in 2023. Reasons: signs of a paper mill; suspected computer-generated content; unreliable results or conclusions; lack of ethics approval or compliance.

## 4. Discussion

Transarterial chemoembolization (TACE) is the most common therapy in unresectable HCC cases [18]. However, due to the presence of portal vein blood supply and abundant collateral circulation in liver cancer tissues, TACE cannot completely inhibit the proliferation of tumor cells. Surviving liver cancer cells will gradually adapt to the hypoxia and ischemia environment, upregulating vascular endothelial growth factor, enhancing angiogenesis, and promoting further tumor invasion and metastasis [19, 20]. Patients treated with TACE require multiple treatments in a short period, resulting in poor quality of life and adverse events. Finding effective chemotherapeutic regimens has become the focus of clinical research [3].

This was the first study to use PSM for comparing the survival of unresectable HCC cases that underwent H101-TACE or cTACE. PSM balanced differences in clinical profiles and risk factors across both cohorts. Otherwise, it would confuse the real effect of H101. In recent years, multiple clinical investigations demonstrated OVs to bring clinical benefits to patients with different types and stages of progression, even metastatic and incurable tumors. More importantly, when combined with chemotherapy, radiotherapy, and immunotherapy, it has a synergistic effect and can sensitize tumor species that respond poorly to immunotherapy drugs such as immune checkpoint inhibitors. Lin et al. [21] have revealed that TACE + H101 contributed considerable survival leverage on comparison with TACE alone among unresectable HCC cases (the median OS: 12.8 months: 11.6 months, *P* = 0.046; the median PFS: 10.49 months: 9.72 months, *P* = 0.044). He and Lin [13] have reported that H101 combined with TACE prolongs survival within HCC cases (median OS of 17 months). This investigation demonstrated that the H101-TACE cohort had survival rates of 22.1 months and 6.5 months of median PFS. The cTACE cohort had a median survival of 13.1 months and 3.3 months of median PFS. Furthermore, following PSM, posttherapeutic survival within the H101-TACE cohort was markedly improved compared to the cTACE cohort. The OS within this study is much longer than Lin et al. [21]. The possible reasons are as follows: first, the number of cases having enlarged tumors/multiple tumors was only 51.4% and 45.9%, but they were much more than 70% and 60% in He et al.'s research. In addition, 30.3% had vascular invasion in the H101-TACE group, while our study had only 5.4%. Second, H101 can reduce liver function injury, not affect the subsequent treatment, and extend the OS. Finally, the current follow-up time is shorter, and the OS is just a preliminary result. These results suggest that H101 is significantly, as the first approved OV drug is modified by deletion of E1B-55KD and E3-19KD gene fragments of human adenovirus type 5 through genetic-engineering technology, which has a unique dual mechanism-precise oncolytic and systemic immunity [22]. No statistically significant variation existed across multiple indexes across the H101-TACE and c-TACE cohorts. But H101-TACE cohort had a significantly higher proportion of fever patients, and its severity increased. Lu et al. [23] found that patients with fever had significantly higher efficacy than those without fever. They also found that transarterial infusion of adenovirus could trigger the host immune system, with activated cell-mediated immunity influencing tumor regression. Most commonly, therapy-linked adverse reaction of H101 is unabiding influenza-type clinical manifestations through muscle soreness and mild pyrexia (38°C) during treatment day [24]. Such pyrexia remains self-limited, and symptoms begin to fall the next day, not requiring treatment. This study further demonstrated that H101-TACE could regulate HCC expansion and gain survival without side effects.

The article "Prognostic Comparison between cTACE and H101-TACE in Unresectable Hepatocellular Carcinoma (HCC): A Propensity-Score Matching Analysis" was retracted in 2023. Reasons: signs of a paper mill; suspected computer-generated content; unreliable results or conclusions; lack of ethics approval or compliance.

The major limitations of the present study were as follows: first, the investigation design was retrospective, and the cohort size was modest, which may cause selection bias. Second, the median follow-up period was relatively reduced, rendering it challenging for thorough OS evaluations. Consequently, future studies employing larger, multicenter cohorts with adequate observational periods are required to validate such outcomes.

## 5. Conclusion

According to the results of the current study, transcatheter H101 treatment combined with TACE can offer enhanced efficacy/tumor response leverage compared to established TACE alone in patients of unresectable HCC.

## Figures and Tables

**Figure 1:** Kaplan–Meier survival curves for OS/PFS within unresectable HCC cases. OS for unresectable HCC patients having H101-TACE and cTACE cohorts (37 cases vs. 74 cases) prior to PSM (a) (*P* = 0.043); PFS within H101-TACE and cTACE cohorts (37 cases vs. 74 cases) prior to PSM (c) (*P* = 0.046); OS for unresectable HCC cases with H101-TACE and cTACE cohorts (36 cases vs. 36 cases) following PSM (b) (*P* = 0.004); PFS within H101-TACE and cTACE cohorts (36 cases vs. 36 cases) following PSM (d) (*P* = 0.012). H101-TACE: transarterial chemoembolization combined with H101; cTAC: conventional transarterial chemoembolization.

The article "Prognostic Comparison between cTACE and H101-TACE in Unresectable Hepatocellular Carcinoma (HCC): A Propensity-Score Matching Analysis" was retracted in 2023. Reasons: signs of a paper mill; suspected computer-generated content; unreliable results or conclusions; lack of ethics approval or compliance.

**Table 1:** Baseline characteristics of the study population before matching.

	H101-TACE (*N* = 37)	c-TACE (*N* = 74)	*P*
Age (years), mean ± SD	57.08 ± 7.68	59.61 ± 9.87	0.172
Gender, *n* (%)			0.108
Male	34 (91.9)	58 (78.4)	
Female	3 (8.1)	16 (21.6)	
HBV, *n* (%)			0.549
Absent	0	3 (4.1)	
Present	37 (100)	71 (95.9)	
ECOG − PS > 0, *n* (%)			0.241
0	29 (78.4)	52 (70.3)	
1	8 (21.6)	19 (25.7)	
2	0	3 (4.1)	
Child-Pugh, *n* (%)			0.834
A	25 (67.6)	48 (64.9)	
B	12 (32.4)	26 (35.1)	
BCLC, *n* (%)			1.000
B	25 (67.6)	50 (67.6)	
C	12 (32.4)	24 (32.4)	
Tumor number, *n* (%)			1.000
≤3	19 (51.4)	38 (51.4)	
>3	18 (48.6)	36 (48.6)	
Tumor size (cm), *n* (%)			0.690
<5	20 (54.1)	43 (58.1)	
≥5	17 (45.9)	31 (41.9)	
Tumor thrombus, *n* (%)			0.136
Absent	35 (94.6)	62 (83.8)	
Present	2 (5.4)	12 (16.2)	
Lymph node metastasis, *n* (%)			0.427
Absent	29 (78.4)	63 (85.1)	
Present	8 (21.6)	11 (14.9)	
Distant metastasis, *n* (%)			0.748
Absent	34 (91.9)	65 (87.8)	
Present	3 (8.1)	9 (12.2)	
Alpha-fetoprotein (ng/ml), *n* (%)			0.408
<400	22 (59.5)	50 (67.6)	
≥ 400	15 (40.5)	24 (32.4)	
TB, mean ± SD	17.69 ± 5.93	16.42 ± 8.97	0.439
ALB, mean ± SD	41.50 ± 4.26	39.76 ± 4.23	0.043
ALT, mean ± SD	34.46 ± 22.71	34.97 ± 32.74	0.932
AST, mean ± SD	33.35 ± 16.35	32.59 ± 22.50	0.856
PT, mean ± SD	13.31 ± 1.26	13.51 ± 1.18	0.411
Ascites, *n* (%)			1.000
Absent	32 (86.5)	64 (86.5)	
Present	5 (13.5)	10 (13.5)	

**Table 2:** Comparison of baseline characteristics between the two cohorts following matching.

	H101-TACE (*N* = 36)	c-TACE (*N* = 36)	*P*
Age (years), mean ± SD	57.03 ± 7.78	57.06 ± 9.82	0.989
Gender, *n* (%)			0.710
Male	33 (91.7)	31 (86.1)	
Female	3 (8.3)	5 (13.9)	
HBV, *n* (%)			1.000
Absent	0	0 (4.1)	
Present	36 (100)	36 (100)	
ECOG − PS > 0, *n* (%)			1.000
0	28 (77.8)	28 (77.8)	
1	8 (22.2)	8 (22.2)	
2	0 (0)	0 (0)	
Child-Pugh, *n* (%)			0.605
A	24 (66.7)	27 (75)	
B	12 (33.3)	9 (25)	
BCLC, *n* (%)			1.000
B	25 (69.4)	25 (69.4)	
C	11 (30.6)	11 (30.6)	
Tumor number, *n* (%)			1.000
≤3	18 (50)	17 (47.2)	
>3	18 (50)	19 (52.8)	
Tumor size (cm), *n* (%)			0.813
<5	19 (52.8)	21 (58.3)	
≥5	17 (47.2)	15 (41.7)	
Tumor thrombus, *n* (%)			1.000
Absent	34 (94.4)	34 (94.4)	
Present	2 (5.6)	2 (5.6)	
Lymph node metastasis, *n* (%)			0.767
Absent	28 (77.8)	30 (83.3)	
Present	8 (22.2)	6 (16.7)	
Distant metastasis, *n* (%)			0.478
Absent	33 (91.7)	30 (83.3)	
Present	3 (8.3)	6 (16.7)	
Alpha-fetoprotein (ng/ml), *n* (%)			1.000
<400	22 (61.1)	22 (61.1)	
≥400	14 (38.9)	14 (38.9)	
TB, mean ± SD	17.80 ± 5.98	14.51 ± 6.33	0.026
ALB, mean ± SD	41.41 ± 4.28	41.30 ± 3.27	0.899
ALT, mean ± SD	34.67 ± 23.00	38.31 ± 41.08	0.644
AST, mean ± SD	33.64 ± 16.48	28.72 ± 13.05	0.165
PT, mean ± SD	13.30 ± 1.28	13.53 ± 1.12	0.421
Ascites, *n* (%)			0.710
Absent	31 (86.1)	33 (91.7)	
Present	5 (13.9)	3 (8.3)	

Abbreviations: ECOG: Eastern Cooperative Oncology Cohort; HBV: hepatitis B virus; BCLC: Barcelona clinic liver cancer; AFP: alpha-fetoprotein; TB: total bilirubin; ALB: albumin; ALT: alanine aminotransferase; AST: aspartate aminotransferase.

The article "Prognostic Comparison between cTACE and H101-TACE in Unresectable Hepatocellular Carcinoma (HCC): A Propensity-Score Matching Analysis" was retracted in 2023. Reasons: signs of a paper mill; suspected computer-generated content; unreliable results or conclusions; lack of ethics approval or compliance.

**Table 3:** Survival prognosis-linked factor assessments.

Factor	Overall survival				Progression-free survival			
	Univariate analysis		Multivariate analysis		Univariate analysis		Multivariate analysis	
	HR (95% CI)	*P*	HR (95% CI)	*P*	HR (95% CI)	*P*	HR (95% CI)	*P*
Sex								
Female/male	1.114 (0.524-2.365)	0.779			0.788 (0.466-1.330)	0.372		
Age (years)								
<60/≥60	0.908 (0.526-1.566)	0.728			0.870 (0.580-1.307)	0.504		
HBsAg								
Positive/negative	0.359 (0.111-1.157)	0.086	0.173 (0.051-0.589)	0.005	0.748 (0.235-2.379)	0.622		
Child-Pugh grade								
B/A	2.018 (1.187-3.433)	0.010			1.082 (0.713-1.643)	0.712		
AFP level (ug/L)								
≥400/<400	2.052 (1.192-3.534)	0.010	1.923 (1.069-3.460)	0.029	1.514 (0.995-2.304)	0.053	1.548 (1.009-2.374)	0.045
Number of tumors								
>3/≤3	0.653 (0.384-1.112)	0.117			1.122 (0.754-1.667)	0.571		
Tumor size (cm)								
≥5/<5	0.888 (0.521-1.515)	0.063			1.178 (0.791-1.754)	0.420		
Tumor thrombus								
Yes/no	6.911 (3.425-13.942)	<0.01	4.944 (2.300-10.628)	<0.01	2.004 (1.083-3.708)	0.027		
Lymph node metastasis								
Yes/no	2.322 (1.211-4.451)	0.011			1.281 (0.758-2.164)	0.356		
Distant metastasis								
Yes/no	1.673 (0.706-3.967)	0.243			1.199 (0.622-2.313)	0.587		
Treatment option								
cTACE/H101-TACE	0.544 (0.300-0.989)	0.046			0.649 (0.423-0.996)	0.048		
BCLC								
C/B	2.999 (1.705-5.272)	<0.01			1.285 (0.834 -1.980)	0.255		
ECOG								
1/0	2.664 (1.520-4.669)	<0.01	2.300 (1.274-4.152)	0.006	1.289 (0.815-2.039)	0.278	1.207 (0.760-1.919)	0.4255
2/0	9.06 (2.673-30.705)	<0.01	7.407 (1.984-27.653)	0.003	9.397 (2.750-32.107)	0.004	10.713 (3.100-37.028)	<0.01

Abbreviations: ECOG: Eastern Cooperative Oncology Cohort; BCLC: Barcelona clinic liver cancer; AFP: alpha-fetoprotein.

**Table 4:** Tumor responses in two cohorts.

	H101-TACE (*n* = 37)	c-TACE (*n* = 74)	*P*
Response			0.025	
CR	6 (16.2)	3 (4.1)		
PR	17 (45.9)	24 (32.4)		
SD	7 (18.9)	17 (23)		
PD	7 (18.9)	30 (40.5)		
ORR	23 (62.2)	27 (36.5)	0.018	
DCR	30 (81.1)	44 (59.5)	0.039	

Abbreviations: CR: complete response; PR: partial response; SD: stable disease; PD: progressive disease; ORR: objective response rate; DCR: disease control rate.

The article "Prognostic Comparison between cTACE and H101-TACE in Unresectable Hepatocellular Carcinoma (HCC): A Propensity-Score Matching Analysis" was retracted in 2023. Reasons: signs of a paper mill; suspected computer-generated content; unreliable results or conclusions; lack of ethics approval or compliance.

**Table 5:** The changes in blood routine and liver function between the two cohorts following operation.

	H101-TACE (*n* = 37)		c-TACE (*n* = 74)	
	3 days following the operation	5 days following the operation	3 days following the operation	5 days following the operation
CRP	64.86 ± 47.23	56.67 ± 48.66	89.96 ± 69.91	76.25 ± 63.75
TB	23.43 ± 11.49	19.44 ± 11.18	28.08 ± 20.23	24.37 ± 15.99
ALB	36.82 ± 3.68	36.55 ± 3.84	35.94 ± 4.10	35.23 ± 3.48
ALT	193.30 ± 196.48	84.81 ± 61.63	135.23 ± 124.90	80.47 ± 57.20
AST	107.05 ± 118.55	36.92 ± 18.13	84.54 ± 69.91	47.23 ± 40.85
WBC	6.28 ± 2.38	7.41 ± 9.57	7.07 ± 3.04	6.20 ± 2.46
PLT	100.78 ± 46.58	115.03 ± 48.36	109.81 ± 53.60	123.26 ± 58.17

Abbreviations: CRP: C-reactive protein; TB: total bilirubin; ALB: albumin; ALT: alanine aminotransferase; AST: aspartate aminotransferase; WBC: white blood cells; PLT: platelets.

**Table 6:** Incidence of postoperative adverse reactions in two cohorts.

	H101-TACE (*n* = 37)	c-TACE (*n* = 74)	*P*
Vomit			0.526	
0	16 (43.2)	24 (32.4)		
1	16 (43.2)	37 (50.0)		
2	5 (16.2)	13 (17.6)		
Abdominal pain			0.185	
0	15 (40.5)	17 (23.0)		
1	13 (35.1)	36 (48.6)		
2	8 (21.6)	15 (20.3)		
3	1 (2.7)	6 (8.1)		
Fever			0.048	
0	4 (10.8)	24 (32.4)		
1	17 (45.9)	32 (43.2)		
2	12 (32.4)	15 (20.3)		
3	4 (10.8)	3 (4.1)		

## Data Availability

Data will be provided upon request to authors.
